# Prevention of tumor risk associated with the reprogramming of human pluripotent stem cells

**DOI:** 10.1186/s13046-020-01584-0

**Published:** 2020-06-03

**Authors:** Kenly Wuputra, Chia-Chen Ku, Deng-Chyang Wu, Ying-Chu Lin, Shigeo Saito, Kazunari K. Yokoyama

**Affiliations:** 1 Graduate Institute of Medicine, Kaohsiung Medical University, 100 Shih-Chuan 1st Rd., San-Ming District Kaohsiung, 807 Taiwan; 2 Regenerative Medicine and Cell Therapy Research Center, Kaohsiung Medical University Hospital, Kaohsiung, 807 Taiwan; 3 Division of Gastroenterology, Department of Internal Medicine, Kaohsiung Medical University Hospital, Kaohsiung, 807 Taiwan; 4 School of Dentistry, School of Medicine, Kaohsiung Medical University, Kaohsiung, 807 Taiwan; 5 Waseda University Research Institute for Science and Engineering, Shinjuku, Tokyo, 162-8480 Japan; 6 Saito Laboratory of Cell Technology Institute, Yaita, Tochigi, 329-1571 Japan

**Keywords:** Cancer risk, Cell reprogramming, Pluripotent stem cells, Regenerative medicine, Therapeutic agents

## Abstract

Human pluripotent embryonic stem cells have two special features: self-renewal and pluripotency. It is important to understand the properties of pluripotent stem cells and reprogrammed stem cells. One of the major problems is the risk of reprogrammed stem cells developing into tumors. To understand the process of differentiation through which stem cells develop into cancer cells, investigators have attempted to identify the key factors that generate tumors in humans. The most effective method for the prevention of tumorigenesis is the exclusion of cancer cells during cell reprogramming. The risk of cancer formation is dependent on mutations of oncogenes and tumor suppressor genes during the conversion of stem cells to cancer cells and on the environmental effects of pluripotent stem cells. Dissecting the processes of epigenetic regulation and chromatin regulation may be helpful for achieving correct cell reprogramming without inducing tumor formation and for developing new drugs for cancer treatment. This review focuses on the risk of tumor formation by human pluripotent stem cells, and on the possible treatment options if it occurs. Potential new techniques that target epigenetic processes and chromatin regulation provide opportunities for human cancer modeling and clinical applications of regenerative medicine.

## Background

The first successful mammalian reprogramming of vegetal cells to totipotent cells using the technology of nuclear transfer generated the cloned sheep “Dolly” [1]. In recent decades, the problems caused by tumorigenesis generated by oocytes (embryos) created by nuclear transfer have been underestimated. The creation of induced pluripotent stem cells (iPSCs) requires the expression of stemness-related genes, such as the combination of *Oct4*, *Sox2*, *Klf4*, and c-*Myc* (OSKM) and that of *Oct4*, *Sox2*, *Nanog* and *Lin28* (OSNL) [2–5]. Studies of the risk of tumorigenesis and cancerous transformation have considered somatic cell reprogramming in the context of cancer patient-specific reprogramming [2–12].

Stem cells are putative candidates for cancerous transformation given their ability to self-renew and to dedifferentiate, which can lead to the acquisition of both the genetic and epigenetic modifications required for tumorigenesis [13, 14]. The stemness-related transcription factors are expressed in embryonic stem cells (ESCs) and adult stem cells, but they are not generally expressed in adult somatic cells. Abnormal expression of ESC-specific factors has recently been reported in human tumors [15–17]. A retrospective study of human patient cohorts has shown that the expression of these factors with survival outcomes in specific tumor types, which suggests that these factors may be useful for assessing patient prognosis [18].

A recent study reported that the clinical expression of the pluripotent factors OCT4, SOX2, and NANOG (OSN) in cancer patients was associated with treatment resistance of lethal cancers [19]. This expression signature was observed in a large cohort of cancers (*n* = 884), comprising renal (*n* = 317), bladder (*n* = 292), and prostate (*n* = 275) cancers. The rates of triple coexpression of OSN were 93, 86, and 54% in prostate, invasive cancer of bladder, and renal cancer, respectively. The high level of expression of OSN was also related to worse prognosis and shorter survival. The major regulators of stem cell pluripotency correlated well with poor survival and treatment resistance of cancer. .

One study showed the production of induced transformed cancer stem cells (CSCs) from differentiated cells [20]. Another study showed that the reprogramming of cancer cells with abnormal or deleted p53 enhanced the generation of pluripotent CSCs and the frequency of tumorigenesis by these reprogrammed CSCs [21]. A reprogramming method has been applied to several types of tumor cells as a possible trial for suppressing tumorigenesis [22–24]. In these studies, some reprogramming factors were delivered to cancerous cells to generate induced pluripotent CSCs (iPCSCs). This method may provide a good model of tumorigenesis and may have therapeutic potential in the prevention of the initiation of carcinogenesis.

In addition to the use of genetic materials to generate pluripotent stem cells, small-molecule compounds that can promote cell reprogramming have also been used to obtain iPSCs. Small molecules that target molecules in signaling pathways, including the inhibition of histone deacetylase (HDAC), Wnt signaling, and transforming growth factor β (TGFβ) can regulate the expression of genes for pluripotent factors, whose expression can lead to the reprogramming of cells [25]. Various molecules that promote cell reprogramming can be used as substitutes for genetic materials. These include recombinant reprogramming factors (e.g., OSKM) modified by a polyarginine [26] and by small-molecule compounds [27–32]. However, the use of chemically defined small molecules alone has not yet generated human iPSCs (hiPSCs) [33]. Furthermore, it has not been clarified whether these small-molecule-driven iPSCs have a reduced risk of tumorigenesis after their therapeutic transfer [34].

In this review, we discuss the current understanding of the risk of tumor formation associated with the reprogramming of various human stem cell-like cells and summarize the possible solutions, such as using anticancer treatments and inhibitors to suppress tumorigenesis in iPSCs, CSCs, and their derivatives (Fig. 1). We have excluded a description of the effects of long noncoding RNAs and microRNAs (miRNAs) on reprogramming in detail from this review article [35, 36].

**Fig. 1:** Schematic representation of the recycling of autologous patient-specific induced pluripotent stem cells (iPSCs) to cure human diseases. Somatic cells from patients are established as patient-specific iPSCs, which are corrected genetically by repairing the defect and then differentiating the corrected iPSCs into autologous progenitor cells for use in transplantation. To correct a gene mutation in patient-specific iPSCs, the genetic code and epigenetic factors are corrected using gene editing, antisense, ribozymes, and peptide nucleic acid (PNA) or modified nucleic acids, and/or chromatin modification

### Characteristics of stem cells and tumor cells

ESCs are established from the inner cell mass (ICM) of blastocyst and can differentiate into all types of cells [15, 16]. The ability to produce teratomas in immune-deficient animals is common pluripotent properties of iPSCs and ESCs [1, 3, 37]. Tumors comprise different types of cancer cells, and this contributes to the heterogeneity of tumors [20]. Teratomas are defined as mixed benign tumors that comprise abnormally developed tissues derived from germ cells with normal karyotypes [37]. Teratomas are regarded as posing no direct danger of forming a malignant tumor, although they have the potential to metastasize in response to some interactions with their microenvironment and niches [38]. Substantial number of tumors can be generated by a series of mutations, which can cause uncontrolled cell division. The process of tumorigenesis is specified by alterations in genetic, epigenetic, cellular, and microenvironmental circumstances [20]. Therefore, the risk of tumorigenesis by any stem cell-derived transplants needs to be eliminated before their clinical applications.

### Stemness-related transcription factors in stem cells and cancer cells

To understand difference between and similarities in marker genes in CSCs and ESCs, we have summarized the corresponding signals and their characteristics (Table 1) [16, 17, 39].

**Table 1:** Summary of the characteristics of embryonic stem cells and cancer stem cells according to theirtranscription factors, markers, signaling pathways, RNA,and epigenetic regulators

Stem cells	ESC		CSC	
Features	mESC	hESC		
Markers [17]	• Oct 3/4 [17] • Sox2 [17] • Nanog [17] • Klf4 [17] • SSEA1 [16] • Esrrb [39]	• Oct 3/4 [17] • Sox2 [17] • Nanog [17] • Klf4 [17] • c-Myc [17] • SSEA3, 4, 5 [16] • TRA-1-60 [16] • TRA-1-81 [16]	• EpCAM (CD326) [17] • Lgr5 [17] • CD19 [17] • CD24 [17] • CD27 [17] • CD38 [17] • CD45 [17] • CD49f [17] • TNFRSF16 [17] • CD133 [17] • CD151 [17] • ABCG2 [17]	• ALDH1A1 [17] • CD13 [17] • CD20 [17] • CD26 [17] • CD34 [17] • CD44 [17] • CD47 [17] • CD66c [17] • CD105 [17] • CD117/c-Kit [17] • CD166 [17]
Signal & Characteristics	• LIF/Jak/Stat (Self-renewal) [40]			
	• Wnt/β-catenin (Self-renewal) [41]	Wnt/β-catenin(self-renewal/Differentiation) [42]	Wnt/β-catenin • Brain [43] • Colon [13] • Prostate [44]	Wnt/β-catenin • Breast [45] • Lung [46] • Head and Neck squamous cell carcinoma [47]
	• Hedgehog (Self-renewal) [48]	• Hedgehog (Differentiation) [49]	Hedgehog • Brain [50] • Pancreas [51]	Hedgehog • Breast [52] • Gastric cancer [53]
	• Notch (Differentiation) [54]	• Notch (Differentiation) [54]	Notch [55] • Brain [56] • Colon [57]	Notch • Breast [58] • Pancreas [59]
	• TGF-β/BMP/Smad (Activin/Nodal→ self-renewal) (BMP → self-renewal) [60]	• TGF-β/BMP/Smad (Activin/Nodal→ self-renewal) (BMP → differentiation) [61]	TGFβ/TβRII, Integrin/FAK • Brain [62] • Skin [63] • Gastrointestinal [64]	TGFβ/TβRII, Integrin/FAK • Breast [65] • Colon [66]
	• FGF (Differentiation) [67]	• FGF (Self-renewal) [68]	FGF-FGFR • Bladder [69] • Breast [70]	FGF-FGFR • Brain [71] • Colon [72]
			PI3K/AkT/mTOR • Neuroblastoma [73] • Ovarian [74] • Glioblastoma [75]	
Related markers • DNA methylation regulator • Chromatin regulator	• DMNT1 (Differentiation) [76] • TET2 (Differentiation) [77] • EZH2 (Self-renewal& pluripotency) [78, 79] • BMI-1 (Self-renewal& pluripotency) [80] • Suz12 (Self-renewal & pluripotency) [78] • MLL1 (Self-renewal & pluripotency) [78]		DNMT1 • Colon [81] TET2 • Breast [82] EZH2 • Breast [83] • Brain [84] • Bone [85] BMI-1 • Esophageal [94] • Laryngeal [95] • Salivary adenoid [96] • Colon [97] • Prostate [86] • Head and neck [87] • Colorectal [88] • Lymphoma [89] Suz12 • Breast [90] MLL1 • Brain [91]	• Breast [92] • Hematomalignancy [93] • Pancreas [83] • Colorectal cancer [88]
RNAs	• Let7 and Lin 28 (Differentiation) [98, 99] • Mir-31 (Differentiation) [100] • Mir-145 (Differentiation) [101]	• Mir-200 family (Differentiation) [102] • LncRNA-ROR (Self-renewal) [103]	Let-7 • Breast [104] Mir-200 family • Breast [105] Mir-34, Mir-34α • Brain [106] • Pancreatic [107] • Colon [108] Mir-145 • Brain [109] LncRNA-ROR • Liver [110]	• Prostate [111] • Gastric [112]
Self-renewal	Yes [113]	Yes [113]	Yes [113]	
DNA repair	Yes [114]	Yes [114]	Altered by adaptation to environments, hypoxia condition and cell cycle [114–117]	
Microenviromental protection by niche from noxious agents	Yes [118]	Yes [118]	Yes [119, 120]	
plasticity	Affected by differentiation and dedifferentiation states [121]		• Epithetical mesenchymal transition can self-renewal acquisition. • Dedifferentiation and mutation accumulation in committed cells [122].	

This table is a modified version of the one published by Hadjimichael et al. [400]. CSC: cancer stem cells; ESCs: embryonic stem cells; *mESCs* Mouse ESCs, *hESCs* Human ESCs.

A few examples are described below.

#### OCT4

Expression of OCT4 is required for the maintenance of ESC characteristics [123]. Oct4-deficient mice do not generate the ICM and thus differentiate into the trophectoderm [123]. In addition, reduced expression of Oct4 in mouse ESC (mESC) caused in the upregulation of trophectoderm genes (e.g., *Cdx29*), whose overexpression leads to differentiation into the primitive endoderm and mesoderm [124]. Under serum-free culture conditions, the forced expression of Oct4 in ESCs promotes neuronal differentiation [125]. High expression level of OCT4 is related to poor prognosis in bladder cancer [126, 127], prostate cancer [128], medulloblastoma [129], esophageal squamous cell carcinoma [130], leukemia, and cancers of the ovaries, testicles, and pancreas [18].

#### SOX2

Expression of Sox2 is detected in ICM and extraembryonic ectoderm of preimplantation blastocysts [131]. Sox2-deficient blastocysts cannot generate a pluripotent ICM. Sox2-deficient mESCs differentiate into trophectoderm, and the overexpression of Oct4 can rescue the pluripotency of Sox2-deficient mESCs [132]. These findings suggest that Sox2 is essential to maintain Oct4 expression. Moreover, the synergistic action of Sox2 and Oct4 in Oct-Sox stem cells-enhancers leads to the regulation of various pluripotent genes, including Oct4, Sox2, and Nanog. In contrast, forced expression of Sox2 in ESCs is reported to lead to their differentiation [133, 134]. This effect was reflected by the reduced expression of pluripotency genes Sox2, Oct4, Nanog, Fgf4, and Utf1 [133] and the induced generation of neuroectoderm, mesoderm and trophectoderm [134]. Increased expression of SOX2 correlates with poor prognosis in stage I lung adenocarcinoma [135], esophageal squamous cell carcinoma [136, 137], gastric carcinoma [138–140], small-cell lung carcinoma [141–143], breast cancer [144], testicular tumors [145], and ovarian carcinoma [146].

#### KLF4

KLF4 is one of the Krűppel-like transcription factors family that are involved in reprogramming. Klf4 is expressed in mESCs and is repressed during differentiation [147]. The RNA interference against Klf4 led to the differentiation of ESCs [148, 149], whereas the forced expression of KLF4 delays the differentiation, increases the expression of OCT4, and stimulates self-renewal ability [150]. Klf4 with Oct4 and Sox2 induces the expression of Lefty1 [151] and Nanog [152], KLF4 is also a prognostic predictor of colon cancer [153] and head neck squamous cell carcinoma [154], and is also detected in leukemia, myeloma, testis cancer [18], early stage breast cancer [155], nasopharyngeal cancer [156], and oral cancer [157].

#### Nanog

In the absence of the leukemia inhibitor factor-signal transducer and activator of transcription (LIF-STAT3) pathway, Nanog is required for the maintenance of ESC properties [158, 159]. Chamber et al. found that expression of Nanog was high in Oct4-knockout embryos, whereas its overexpression did not counteract the differentiation program of ESCs induced by Oct4 deletion [159]. In the absence of Nanog, embryos did not produce a pluripotent ICM, but Nanog deficient mESCs could be established [158, 160]. Nanog downregulation in human ESCs promotes differentiation toward the extraembryonic lineage, as demonstrated by the forced expression of endodermal and trophectodermal specific genes. OCT4–SOX2 heterodimer complex binds to the Octamer–Sox *cis*-elements in the proximal promoter of *NANOG* gene and regulate NANOG expression in ESCs [161]. Moreover, Nanog, Oct4, and Sox 2 cooperate with the signaling pathway mediators, which means that signals are delivered directly to the genes regulated by the core factors [162]. Higher expression of NANOG is concerned with poor prognosis for testicular cancer [163], colorectal cancer [164], gastric cancer [140], non-small cell lung carcinoma [165, 166], ovarian cancer [167], and liver cancer [168].

#### C-Myc

c-Myc is one of the factors for stem cell pluripotency, proliferation, and apoptosis [169–171]. c-Myc is directly regulated by LIF-STAT3 signaling, and its constitutive expression renders ESC self-renewal independent of LIF. However, the forced expression of dominant-negative c-Myc induces differentiation [172]. It has been reported that c-Myc represses signaling of the mitogen-activated protein kinase (MAPK) pathway, which led to the inhibition of differentiation [173]. c-Myc binds and regulates the transcription of at least 8000 genes in ESCs including those for E2F–Max complexes, and NuA4 HAT complex, which regulate ESC pluripotency [174]. c-Myc was one of the most important leukemia stemness factors. C-MYC overexpression is found in over 70% of human cancers, including breast cancer, colon cancer, glioma, medulloblastoma, pancreatic cancer, and prostate cancer [18, 175]. c-MYC expression correlates with poor prognosis for hepatocellular carcinoma [176] and early carcinoma of the uterine cervix [177, 178]. c-MYC-driven reprogramming is controlled by the activation of c-MYC-mediated oncogenic enhancers in human mammary epithelial cells [179].

#### p53

The inhibition of the tumor suppressor protein 53 (TP53) increases the rate of reprogramming of fibroblasts to iPSCs [180, 181], which can differentiate into dopaminergic neurons directly from human fibroblasts [182].

#### JDP2

The c-Jun dimerization protein 2 (JDP2) is a member of the AP-1/ATF family of transcription factors and can function as a histone chaperone that regulates transcription [183–185]. JDP2 is a reprogramming factor because it can regulate the Wnt signaling and function as a suppressor of producing reactive oxygen species (ROS) [186–189]. For example, addition of the ROS scavenger vitamin C to the culture medium significantly increases the reprogramming efficiency of cultured cells [190]. Activation of the Wnt signaling can maintain the ability for pluripotency in ESCs [41, 191–194]. ESCs can differentiate into all types of cells, except for some in extraembryonic tissues [37, 38]. The cell reprogramming method that uses OCT4 and JDP2 to generate gastric cancer cells is based on this notion [195]. In that study, reprogramming using these two factors inhibited the tumorigenic function of gastric cancer cells by inhibiting bone morphogenetic protein 7 (BMP7). Moreover, reprogrammed gastric CSC-like cells induced a lower level of tumor formation in immune-deficient mice than did the parental cancer cells [195]. This method is a good example of a therapeutic strategy that might restrict cancer progression by using JDP2 together with OCT4 as reprogramming factors. Collectively, accumulating evidence suggests that ESCs and CSCs share major transcription factors.

### Surface markers for stemness in CSCs

The uncontrolled proliferation of many tumors is driven by a small population of cancer cells, known as CSCs, which exhibit the capacity for self-renewal and pluripotency. Unlike somatic cancer cells, CSCs can produce an obvious cancer and propagate the malignant cancerous clones indefinitely. Like the stemness-related transcription factors, surface markers that are expressed in stem cells are also expressed in human cancers. These include TRA-1-60, Stage specific embryonic antigen-1(SSEA-1), Epithelial cell adhesion molecule (EpCAM), Aldehyde dehydrogenase 1 family, member A1 (ALDH1A1), Leucine-rich repeat-containing G-protein coupled receptor 5 (Lgr5), CD13, CD19, CD20, CD24, CD27, CD34, CD44, CD45, CD47, CD49f, CD66c, CD90, CD166, TNFRSF16, CD105, CD133, c-Kit, CD138, CD151, and CD166. Table 1 shows the surface markers of CSCs, some of which are targets of therapeutics in cancer treatment.

#### CD133

CD133 is a transmembrane glycoprotein that localizes to cellular protrusions. It is originally known as a stem cell marker which is detected in neuroepithelial stem cells [196] and has been recognized as a CSC marker [197]. This molecule is used to identify many different types of CSCs, including those originating from glioma [198], and colorectal [199, 200], lung [201], liver [202], and prostate [203] cancers. CD133 has been shown to be involved in the regulation of glucose uptake and glucosamine production under condition of high-glucose, circumstances related to glycolysis, and autophagy [204]. However, knockdown of CD133 has no significant effect on cancer development [205]. Both CD133+ and CD133– metastatic colon cancer cells are initiated equally during the early stage of tumor formation [206], which indicates that CD133 expression is not specific and not restricted to stem cells. Therefore, CD133 seems to reflect glucose availability and is not a specific marker of CSCs.

#### CD44

CD44 is another transmembrane glycoprotein. CD44 is concerned with cell division, migration, and adhesion via different signaling [207]. It is expressed in both normal fetal and adult hematopoietic stem cells. Upon binding to hyaluronic acid (HA), its primary ligand, CD44 mediates cell-cell communication and signal transaction. HA binding to CD44 on cell surface molecules, such as selectin, collagen, osteopontin, fibronectin, and laminin, activates the epidermal growth factor receptor tyrosine kinase and increases cell proliferation and survival through the signals of MAPK and phosphatidylinositol-3-kinase (PI3K)-Akt pathways [208, 209]. Knockdown of CD44 prevents the tumors occurrence induced by colorectal CSCs [205]. CD44 plays a role in in the invasive and tumorigenic abilities with stemness features of several tumor cell types, including breast [210, 211], prostate [212, 213], colon [214, 215], and pancreas [216] cancers, and head and neck squamous carcinoma [217]. Therefore, CD44 is not specific for CSCs but is more of a marker of invasive or metastatic cells. Several other CSC surface markers appear to function in specific types of tumors.

#### ABCG2

ABCG2 is one of the ATP-binding cassette transporter (ABC) family. ABCG2 may be a universal biomarker of stem cells [16]. ABCG2 plays a vital role in stimulating the proliferation of stem cells and, in the case of esophageal squamous carcinoma, has been shown to be required for the maintenance of the stem cell phenotype [218]. The sensitivity of hepatocarcinoma cells to the chemotherapeutic drugs, doxorubicin and 5-fluorouracil, correlates inversely with the surface levels of AGCG2. The AGCG2 level expressed on cancer cells, including colon cancer lines, also correlates closely with tumorigenicity, drug resistance, proliferation, and metastatic ability [219, 220].

#### CD13

CD13 encodes the enzyme aminopeptidase N, a Zn2 + −dependent membrane-bound ectopeptidase. CD13 is overexpressed in multiple cancers, including hepatocarcinoma [221], and colon cancer [222], as well as on the surface of vasculature endothelial cells in tumors undergoing angiogenesis [223].

#### Lgr5

Lgr5 is one of the leucine-rich repeat-containing G-protein-coupled receptor (GPR49) family, which belongs to the seven-transmembrane G-protein-coupled receptor super family. Lgr1 ~ 5 family members are regulatory receptors involved in Wnt signaling [224]. Lgr5 binds to the furin-like repeat domains of R-spondin 1 ~ 4 (RSPO1 ~ 4) to potentiate WNT signaling [225]. However, RSPO1–Lgr5 can also directly activate TGFβ signaling in a cooperative interaction with the TGFβ type II receptor on colon cancer cells, which increases growth inhibition and apoptosis [226]. The effect of Lgr5 expression depends on its interactions with the both Wnt and TGFβ signaling systems [227]. Lgr5 is expressed in many organs including the brain, mammary glands, intestinal tract, stomach, hair follicles, eyes, and reproductive organs [226]. Lgr5 is also a Wnt signaling target. Its expression I increased in prostaglandin E2 (PGE2)-treated colorectal cancer cell lines, but Lgr5 knockdown inhibits the PGE2 survival response and increases cell death [224]. Lgr5 seems to be a global marker of adult stem cells, such as those found in the hair follicles, intestine, liver, colon, rectum, and ovaries [228], and a definitive surface marker of colorectal CSCs that is coexpressed with CD44 and EpCAM [229].

#### CD326 (EpCAM)

The surface marker EpCAM is a type I transmembrane glycoprotein that acts as a calcium-independent homophilic adhesion receptor with a molecular weight 30–40 kDa. EpCAM is expressed in epithelial tissues, progenitor cells, cancer cells, and stem and germ cells [230]. EpCAM can be downregulated when cancer cells undergo the epithelial-mesenchymal transition (EMT). The wide distribution of EpCAM expression on most cancer cells indicates that it is not a specific marker of CSCs [231].

### Stemness-related signaling pathways

Three processes such as maintenance, self-renewal, and differentiation are concerned with embryonic development and homeostasis of adult tissues. Cancers commonly exhibit aberrant functions within these pathways, often in a cell context-dependent manner. Here we discuss the current evidence for the control of the Hedghog (Hh), Notch, LIF-JAK-STAT, PI3K-Akt-mammalian target of rapamycin (mTOR) and Wnt/β-Catenin pathways in CSCs.

#### Hh signaling

The Hh ligands (Desert hedgehog, Sonic hedgehog, and Indian hedgehog) bind to Patched, which activates downstream signals that lead to the nuclear localization of transcription factors, followed by the upregulation of genes involved in survival, proliferation, and angiogenesis [232]. Hh is the major regulator of vertebrate embryo development, stem cell maintenance, cell growth and differentiation, tissue polarity, cell proliferation, and the EMT [233]. Hh signaling is implicated in CSC self-renewal and cell-fate determination [232] and is considered as a potential therapeutic target in the treatment of breast cancer and pancreatic cancers [234].

#### Notch signaling

Notch is controlled with cell–cell communication through transmembrane receptors and ligands. In human ESCs, Notch signaling governs the cell-fate determination in the developing embryos and is required for the development of all three germ layers from undifferentiated ESCs [235]. In CSCs, Notch controls tumor immunity and CSC maintenance [59]. Notch signaling is frequently dysregulated in cancers, which provides a survival advantage for tumors and a potential target in the treatment of cancers [236].

#### LIF–JAK–STAT signaling

LIF–JAK–STAT signaling governs the cell-fate determination, is important in cytokine-mediated immune responses, and is involved in many biological processes such as proliferation, apoptosis, migration, and stem cell regulation [237]. Tight control of JAK–STAT signaling is required for maintenance of stem cells, self-renewal, and anchoring of stem cells in their respective niches by through the regulation of different adhesion molecules.

#### PI3K–Akt–mTOR signaling

PI3K–Akt–mTOR signaling is crucial to stem cell proliferation, metabolism, and differentiation. This pathway may dysregulate in human cancers [238]. Over 70% of ovarian cancer cells is reported to activate PI3K–Akt–mTOR pathway. This pathway is a therapeutic target in the treatment of this cancer type [74] as well as for neuroblastoma [239], endometrial cancer [239], and acute myeloid leukemia [240].

#### Wnt–βcatenin signaling

Wnt signaling plays a role in the stem cell differentiation, and dysregulation of Wnt signaling is associated with the expansion of stem and/or progenitor cells, as well as carcinogenesis [241], Targeting of Wnt is one treatment option for hematological malignancies [242], liver cancer [243], and other types of tumors [244].

### Mutation of the genome

The first event that triggers the transformation of normal cells into abnormal cells is mutation of the genome. Such mutations may be maintained, and other events, such as changes in the epigenome of stemness-related genes, oncogenes, and tumor suppressor genes, can also trigger the transformation into abnormal cells.

In general, “driver” mutations occur during the initiation stage of cancer and are followed by the accumulation of “passenger” mutations and tumorigenesis [245, 246]. Driver mutations trigger the growth and development of cancers, whereas passenger mutations do not affect clonality [247–249]. Recent progress in the technology of deep sequencing has led to identify these mutations in particular oncogenes and/or tumor suppressor genes [250]. However, whether these mutations can become a barrier to the reprogramming of cancer cells remains unclear. Moreover, the reprogramming of cancer cells may induce genomic changes, including chromosomal aberrations, copy number variations (CNVs), and single-nucleotide variations. For example, chromosome abbreviations at trisomy 12, chromosome 8, and chromosome X have been found in ESCs and iPSCs [251–256]. CNVs have been detected during reprogramming or mosaicism from parental cells. In some cases, CNVs are also lost by passaging of cells [254, 257–260].

Single-nucleotide mutations have been analyzed using high-throughput next-generation sequencing technologies [261, 262]. Additional investigation is required to characterize the occurrence of these mutations during cell reprogramming. Mutations in mitochondrial DNA in human iPSCs increase with age, and the use of young donor cells may be one option to overcome this problem [263, 264].

### Epigenetic alterations

The oncogenic potential of reprogrammed stem cells correlates with epigenetic and genomic instability [265, 266]. Epigenetic instability during cancer progression can lead to commitment to altered gene expression. Tumor generation can be caused by epigenetic reprogramming such as carcinogenic enhancer reactivation in both somatic and cancer cells [267–269]. In general, DNA methylation can silence the expression of the tumor suppressor genes that are required for sustaining normal function, whereas aberrant expression of oncogenes can lead to cancer initiation [270–272]. Intriguingly, iPSCs generated from human sarcoma cell lines have the same methylation and demethylation status in the promoters of oncogenes and tumor suppressor genes in the initial stages. In some cases, iPSCs can suppress the oncogenic promoters and maintain the activity of the promoter of tumor suppressor genes. These finding suggest that stem cell factors can inhibit the expression of cancer phenotypes, perturb epigenetics, and change cancer-related gene expression [266].

The factors that regulate chromatin are another possible target for circumventing the cancer risk during cellular reprogramming. Histone modification, noncoding RNA alteration, and chromatin alteration around mutated regions of DNA are key events that change oncogenic features [273]. Moreover, recent evidence of super-enhancers, locus control regions, and phase separation has provided new targets for next-generation reprogramming, to limit the oncogenic risk associated with cell reprogramming [273–275]. The methodologies chosen to induce these epigenetic and chromatin changes require careful consideration.

### Epigenetic modifiers and cancer cell plasticity

The differences between CSCs and adult stem cells in the early stage are reflected in differences in stemness signals, such as BMP, notch receptor 1 (Notch 1), sonic hedgehog (Shh) signaling molecule, TGFβ, and the wingless-type MMTV integration site family (Wnt). Later, EMT factors such as HIFs, the zinc-finger protein SNAI2 (Slug), the zinc finger protein SNAI1 (Snail), the class A basic helix–loop–helix protein 38 (Twist 1), and the zinc-finger E-box-binding homeobox 1/2 (Zeb 1/2) are activated, which leads to changes in epigenetic signatures during progression. Changes in the epigenetic machinery might be crucial for the acquisition of stemness characteristics by, and the tumorigenesis of CSCs [276].

The epigenetic barriers that determine cell plasticity must be overcome during the initial steps of cell reprogramming. In the first step, DNA methylation by DNA methyltransferases (DNMTs) occurs at CpG islands and is reversed by ten-eleven translocation proteins (TETs), followed by transcriptional silencing. Both DNMTs and TETs affect transcriptional initiation, elongation, splicing, and stability at the CpG-poor and repeat-rich intergenic loci of target genes [277]. Some methylated DNA-specific binding proteins also perform similar functions. In the second step, histone modifications, such as methylation, acetylation, ubiquitination, phosphorylation, and SUMOylation, cause changes in nucleosomes. These changes define functional regions such as promoters, enhancers, and insulators, which determine the transcriptional patterns and cell fates. In the third step, histone modifiers are used to control chromatin during transcription, replication, and genome maintenance.

Several histone modifiers can regulate transcription, such as the polycomb repressive complex (PRC) 1 and 2, and the enhancer of zeste homolog 2 (EZH2), which is the catalytic subunit of PRC2 that mediates transcriptional repression by introducing H3K27me3 [278]. By contrast, in glioblastomas, the H3K27M mutation in H3.1 and H3.3 leads to reduced EZH2 activity and a decreased level of H3K27me3, followed by a more primitive stem-like state [279, 280]. Loss of EZH2 function can induce a transcription program for self-renewal and leukemogenesis [281]. Therefore, EZH2 mutation and deregulation of H3K27me3 seem to be linked.

The trithorax group (TrxG) complex is another factor that plays a role in the control of histone methyltransferase (HMT) in mixed-lineage leukemia (MLL) [282]. In this type of leukemia, the MLL fusion protein MLL-AF9, which lacks the catalytic domain, is produced by chromosomal rearrangement. The committed cells can be reprogrammed toward leukemic stem cells and initiate tumorigenesis [283]. MLL oncogenic fusion proteins require the repressive activity of PRC1, which mono-ubiquitinates histone H2A at lysine 119 (H2AK119Ubi) and mediates transcriptional repression in association with PRC2 [283]. BMI-1 in PRC1 is required to abolish tumor suppressor functions and to enhance CSC self-renewal in solid tumors [284]. Finally, ATP-dependent chromatin modeling complexes that move, eject, or restructure chromatin, are also key elements in the control of tumorigenesis.

Four subfamilies are involved in chromatin remodeling in tumor cells, such as switch/sucrose nonfermentable (SWI/SNF), imitation switch, chromodomain helicase DNA binding protein 1, and INO80 complex ATPase subunit. These differ in their functions, protein domains, and subunit constituents [285]. Loss of SWI/SNF-related matrix-associated actin-dependent regulator of chromatin subfamily B member 1, a subunit component of the SWI/SNF complex, results in genetic changes that drive rhabdoid tumors and are associated with the inhibition of differentiation, which leads to reprogramming toward oncogenic transcription for oncogenic signaling [286, 287]. The AT-rich interactive domain-containing protein 1A, another subunit of the SWI/SNF complex, functions as a tumor suppressor in colon cancers, and its deletion causes activation of the oncogenic transcriptional program for the promotion of invasive colon adenocarcinoma [288]. These data indicate that epigenetic modifiers also play a critical role in determining stemness/pluripotency and tumorigenesis.

Reversible epigenetic changes play a critical role in the fate decision in cancer cells, which can favor or disfavor the stem cell program that sustains tumor progression. Similarly, cell reprogramming involving epigenesis in cancer cells can generate iPSCs. Chromatin regulators such as the complex of PGC and TrxG proteins can regulate cancers and reprogramming [289]. In glioblastomas, several PRC and TrxG components play important roles in CSC development and in the plasticity of cancer cells. In adult glioblastoma, overexpressed MLL5 represses the expression of H3.3 in CSCs, which causes local reorganization of chromosomes [290]. The upregulation of MLL5 in non-stem cancer cells induces cell plasticity by inhibiting pro-neural differentiation, thereby eliciting a stem cell-like stage.

Another chromatin modifier, the linker histone variant H1.0, is also critical for the plasticity of cancer cells. Perturbation of H1.0 levels affects self-renewal activity directly and promotes the differentiation of non-stem cancer cells, thus blocking their tumorigenicity in vivo [291]. The plasticity of CSCs can be counteracted by epigenetic barriers that prevent cell reprogramming in vitro, such as the deposition of Suv39h1-associated H3K9me2/3 modifications [292]. An interesting insight into these epigenetic barriers was provided by a comparison of the epigenetics of gene expression between adult cells and CSCs in response to tissue damage [293]. In that report, tissue damage activated the resident stem cells, and CSCs exhibited overactivated stress-dependent enhancers and epigenetic modifications, which altered their cell fate and plasticity. These findings highlight the critical role of the reversibility of changes in the chromatin structure in the determination of the functional properties of CSCs.

### Alteration in the microenvironment during tumorigenesis

The tumor microenvironment favors a stress-responsive enhancer, which may induce CSC plasticity. Therefore, the microenvironment and niche seem to be critical for the reprogramming to CSCs and iPSCs. Inflammation is an immune reaction to a pathogen [294], during which the responses of immune cells can lead to oxidative damage of DNA in infected cells. Nuclear factor kB and STAT3 can cause parenchymal cells to produce excess amounts of ROS and reactive nitrogen species, which can induce genomic instability and DNA mutations [295]. Mutations and chromosomal alterations are thought to be associated with tumor progression, which may be potentiated by a chronic inflammatory microenvironment that are damaged by mutations.

During CSCs have developed, CSCs may create their own niche. Cells forming the CSC niche necessary for both the maintenance of CSCs and the generation of factors and tumor-associated cells that maintain CSC properties such as invasion, metastasis, and promotion of angiogenesis [296]. The CSCs niche contains cellular components such as cancer-associated fibroblasts [297], tumor-associated macrophages [298], tumor-associated neutrophils [299], mesenchymal-associated cells [300], and cell-mediated adhesion and soluble factors [301], which played important roles in cell–cell communication.

### How to avoid tumorigenesis in human pluripotent stem cells

Tumor suppressor genes are mostly transcription factors that modulate the antiproliferation signals that arrest the consistency of the cell cycle for DNA repair and that prevent mutation during cell division [302–306]. For example, the p53 tumor suppressor gene protein product functions as a transcription factor and a cytoplasmic regulator in cell cycle arrest and apoptosis [306–308]. The dysregulation of genes that modulate the cell cycle results in uncontrolled cell division, during which a series of mutations to proto-oncogenes and tumor suppressors are needed before cells transform to cancerous cells [309]. Proto-oncogenes are quiescent counterparts of oncogenes that become oncogenes upon mutation. The modified cells produce more of the gene product and exhibit excessive proliferative ability. Hormones or signal transduction can stimulate oncogenes to promote uncontrolled cell proliferation by changing the regulation of gene transcription [310, 311].

Pluripotent reprogramming factors are overexpressed in various cancers [312, 313]. OCT4 has been reported to be overexpressed in a gastric cell line [18], ovarian carcinoma, pancreatic cancer [18], prostate cancer [314], and bladder cancer [315]. c-MYC is also overexpressed in various cancers [316, 317] and can block differentiation and induce tumor formation in the absence of p53 [318, 319]. These observations indicate that reprogramming factors can act as potential proto-oncogenes in the reprogramming process and emphasize the potential risk of carcinogenesis by stem cell-like cells.

### Reprogramming

Reprogramming protocols have been used to inhibit the tumorigenesis induced during reprogramming in studies of various cancer cells [20–22]. In these models, one or multiple sets of reprogramming factors are delivered to cancer cells and induced patient specific CSCs are generated. These models can be used to study therapeutic targets in the initial stage of carcinogenesis [20–22]. In addition to the genetic methods that are used to generate pluripotent stem cells, some small molecules have been reported to promote cell reprogramming. For example, targeting signaling pathways like the HDAC, Wnt, and TGFβ cascades can regulate the expression of pluripotent stemness genes induce the reprogramming of cells [25]. Various molecules that promote reprogramming can replace genetic methods; these include recombinant reprogramming factors (OSKM) with polyarginine tags [26] and other small molecules [30–33]. However, chemically defined small molecules that induce reprogramming alone have not been developed for human induced pluripotent stem cells (hiPSCs) [24]. Furthermore, whether small molecule-driven iPSCs can prevent the risk of tumorigenesis when used therapeutically has not been determined. The ability of undifferentiated iPSCs to produce teratomas in grafted cell populations is one of the main concerns of this approach, and the nature of these cells should be clarified genetically. Precise information about these transplantation animal models, inoculated patient-specific iPSCs, and the resultant organoids is needed.

### Reversibility of the epigenetic state

The use of clones that have been pre-evaluated as being safe is one possibility for overcoming carcinogenic activity, as demonstrated in neural stem cells (NSCs) [320–322]. An antibody against SSEA-5 on human ESCs (hESCs) can be utilized to remove teratoma-forming cells from dissociated hESCs [323]. In immune-deficient mice, flow cytometric analysis has shown that transplants of SSEA-5-negative cells formed smaller teratomas, measuring < 1 cm^3^, whereas SSEA-5-positive transplanted cells formed teratomas > 1 cm^3^. Flow cytometric analysis using an anti-SSEA-5 antibody may be useful for separating undifferentiated, unsafe cells from iPSC-driven mixed-cell populations. The induction of senescence generated by replication stress and DNA damage, telomere shortening, environmental and oncogenic stresses, and the pro- inflammation inducing microenvironments is one of the oncogene-associated events involving epigenetic control [285]. Cancer-associated senescence has been reported to promote cancer stemness and plasticity in CSCs [306].

### Risk management to prevent tumorigenesis

Three different approaches for the removal of tumor-initiating pluripotent stem cells from ESCs and their differentiated cells have been reported: (i) chemical treatment [324–327], (ii) genetic treatment [328–330], and (iii) immunological treatment [323, 331–335] (Table 2). Each method has its advantages and disadvantages; the latter include the high cost, variation between lots, nonspecific antibody binding, integration of toxic genes, and long duration [354]. A strategy for application to clinics to abate the teratoma formation should be explored further [354, 355]. The use of small molecules has several advantages, such as robustness, efficiency, speed, simplicity, and low cost. Some small molecules can inhibit the formation of teratoma in human pluripotent stem cells (hPSCs). For example, an inhibitor of stearoyl-CoA desaturase (SCD), PluriSIns #1, has been shown to prevent teratoma formation [325]. SCD1 is an important enzyme in the biochemical synthesis of monosaturated fatty acids, which are needed for the survival of hPSCs. A recent study reported that SCDs play a critical role in endoplasmic reticulum (ER) stress and promote the survival of glioblastoma cancer stem cells [356]. The N-benzylnonanamide JC101 induces ER stress via the protein kinase RNA-like endoplasmic reticulum kinase/ATF4/DNA damage inducible transcript 3 (DDIT3 = CHOP) pathway [340], which leads to the inhibition of teratoma formation. In a study that used iPSCs to treat spinal cord injury, these cells were determined to be safe before the grafting of transplants, which prevented the formation of teratomas [357].

**Table 2:** Summary of the procedures for reprogramming and the targeted functions in human pluripotent stem cells and their derivatives

Cell Types	Method	Function targeted	Status of tumorigenesis	Tumor treatment	Clinical trail	References
**A. Chemical treatments**						
hPSCs	Inhibitors of stearoyl-CoA desaturase (SCD)1	Oleate = decreased Stearate and Palmitate = increased	Prevent teratoma	Teratoma	(No trial yet)	2013 [325]
ESCs and EBCs	(N-oleoyl serinol) = ceramide analogue	S18	OCT4 (+) / Prostate apoptosis response-4 (PAR-4) (+) = elimination	Human cancer cell lines Brain tumor cell lines Adenocarcinoma cell lines Hepatocarcinoma cell lines	–	2002 [336] 2003 [337]
hESCs	MitoBlock-6	Inhibit ERV/ALR (sulfhydroxyl oxidase)	Impairs import of Mila40/Erv1 and TIM22 Block the teratoma formation	Teratoma	–	2013 [326]
hPSCs, HiPSCs	*Clostridium perfringens* endotoxin (CPE)	Bound several Claudins including Claugin-6	Elimination of tumorigenic PSCs	Teratoma	–	2013 [333]
hESCs, hiPSC-derived cells	Survivin inhibitor (Quercetin or YM155)	Cell death of undifferentiated stem cells, mitochondrial accumulation of p53	Prevent teratoma formation	Gastric cancer	–	2017 [338]
hESCs	Digoxin and Lanatoside C	Cytotoxicity in undifferentiated hESCs	Tumor prevention in hESCs	Teratoma	–	2017 [339]
hESCs	JCO11	ER stress; PERK/AT4/DDIT3 pathway	Inhibition of teratoma formation	Teratoma	–	2014 [340]
**B. Immunological treatment**						
hPSCs	Anti-Claudin 6 (CLDN-6), Anti-CLDN-6 (+) cells removal, Anti-CLODN-6-Cytotoxic Ab, Anti-CLODN-6-Toxin CPE	Decrease the teratoma-formation	Inhibition of Teratoma	Teratoma	–	2013 [333]
hPSCs	Anti-SSEA-5	H-type-1 glycan surface markers, SSEA-5-CD9, CD30, CD50, CD90 and CD200	Removal of cells with teratoma-potential from incompletely differentiated hESCs	Teratoma	–	2011 [323]
hPSCs	UEA-1+ and SSEA-4+	Fut1 and Fut 2 (fucosyl transferases)	Enrichment of PSCs	Teratoma	–	2011 [341]
hESCs	mAb 84 cytotoxic antibody(Podocalyxin-like protein 1)	Kill undifferentiated hSCs	Removal of teratoma formation	Teratoma	–	2009 [331] 2008 [332]
HPSCs derived neural precursor cells	Tra-1-60 (−), Tra-1-81 (−)	Removal of undifferentiated cells by Ab-nanogold	Inhibition of teratoma formation	Teratoma	–	2010 [342]
**C. Genetic treatment**						
hESCs	Survivin (BIRC5), YM155	Apoptosis in hESCs and teratoma formation	Removal of teratoma formation	Teratoma	–	2009 [328]
hESCs	HSV-tk + cells were killed by ganciclovir	Kill HSV-tk (+) cells	Remove the tumor forming cells	HSV-tk + teratoma	–	2003 [330]
hESCs	Nanog-3′ untranslated region with HSV-tk (+) gene	Kill HSV^tk (+) cells	Remove the tumor forming cells	Teratoma	–	2012 [343]
Gastric cancer cells	Overexpression of JDP2, Oct4	BMP7 inhibition	Decreasing teratoma development	Gastric cancer	–	2017 [195]
Neural cells from iPSCs	Pre-evaluation by transfer of iPSCs derived cells to primates	Pre-evaluation of tumor development	No tumor development	Spinal cord injury in marmoset model	–	2012 [344]
Neural cells from iPSCs	Methylation analysis of iPSCs derived cells	Non-methylation status of CAT, PSMD5 genes	No tumor development	Nerval stem progenitors	hiPSC-NS/DCs in clinical model	2017 [303]
Prostate cancer cells	Knock down of Oct4, Sox2	Tumor development screening after in vivo transfer	No tumor development	Prostate cancer DU145.DC3	–	2010 [314]
Cardiac progenitor cells from iPSCs	Inhibitors of DNA topoisomerase	Decreasing teratoma formation	Decreasing teratomas	Teratoma	iPSC-derivet cardiac regenerations	2014 [345]
ES cells	CDK1 inhibitor treatment	Activation of p53-HOXA-MCL1 axis	Prevention of teratoma formation	Teratoma	–	2015 [346]
iPSCs	Inhibition of anti-apoptotic factor, treatment Survivin (YM155)	Pre-evaluation of tumor development	No teratoma formation in mice	Teratoma	–	2017 [347]
iPSCs	Introduction of suicide gene Caspase-9	Pre-evaluation of tumorigenic transformation	Avoid tumorigenic transformation	Injured spial cord of NOD/SCID mice	hiPS/NS/DCs in animal model	2017 [348] 2012 [344]
Neuro-spheres from iPSCs	Pre-evaluation by transfer of iPSCs derived cells to mice	Pre-evaluation of tumor development	No tumor development	Spinal cord injury (SCI) patients tratment in animal model	hiPS/NS/DCs in animal model	2011 [349]
Pancreatic ductal adenocarcinoma derived PDAC	* Tet-OSKM & MzrtTA * Mir302-OCT4 * Episomal vector	Reduced tumorgenicity TET2, SirT1, and Dot1L were decreased. TET1 upregulated & Tbx downregulated	Nanog is required. Tra-1-80 decreased	Reprogrammed pancreatic ductal adenocarcinoma (PDAC)-Tumergenesis	–	2019 [350]
Ischemic Cardiomyopathy cells	EZH2, FoxM1 epigenetic repressed in PRC2 KLF15 decreased	DNA methylation on targetsof KLF15 Epigenetic regulator suppressed metabolic reprogramming of ICM	KLF15 repression	Ischemic cardiomyopathy (ICM)-Reprogramming	–	2019 [351]
Ovarian cancer cells	C/EBPBeta-DOT1L	Open chromatin	H3K79 methylation	Ovarian cancer cells-Reprogramming	–	2018 [352]
Pediatric cancer derived iPSCs	Dnmt3a ablation	De novo ICR-preferred CGI hypermethylation ICR-CpG islands	Cancer repressed	In vivo pluripotency	–	2017 [353]

The introduction of inhibitors of antiapoptotic factors that effectively remove residual iPSCs can also prevent teratoma formation [344, 348]. Treatment with survivin (an antiapoptotic factor) and a novel survivin suppressant, YM155, was effective in decreasing the risk of teratoma formation. In that study, addition of YM155 permitted the survival of CD34^+^ cord blood cells and prevented teratoma formation in human induced pluripotent stem cells (hiPSCs)-grafted mice [347].

The introduction of inducible caspase-9 (iCap9), as a suicide gene, into hiPSCs avoided tumorigenic transformation after their transplantation [347, 348]. The efficiency of iCap9 and small molecule-like chemically induced dimerization (CID) in the prevention of the risk of tumorigenesis was evaluated in cell-transplantation experiments. iCap9 integrated with CID induced the apoptosis of iPSCs and iPSC-derived NSCs and produced the terminal differentiation of transduced cells grafted into injured spinal cord in mice but avoided the formation of teratomas [348].

A conditionally replicating adenovirus that targets cancers using multiple factors (m-CRAs) is a new antitumorigenic agent used in hPSC-based cell therapy. Given that the survivin promoter is stronger in undifferentiated hPSCs than was the telomerase reverse transcriptase (TERT) promoter, surviving promoter m-CRAs efficiently kill undifferentiated hPSCs but not differentiated normal cells when compared with TERT promoter m-CRAs. The surviving promoter m-CRAs seems to be a novel antitumorigenic agent that may facilitate safer hPSC-based medical applications [358].

Another approach is the isolation of the desired differentiated cells from other cell types and undifferentiated hPSCs, such as the removal method of the residual pluripotent cells from other cells using fluorescence-activated cell sorting or antibodies coated magnetic beads against a particular antigen, including SSEA-5 [323], claudin-6 [333, 359], and the *Ulex europaeus* agglutinin-1 fucose-binding lectin (UEA) [360]. Caludin-6 bound to the enterotoxin produced by *Clostridium perfringens* kills the hPSCs that induce teratoma formation [333]. Yet another approach is the direct, targeted killing of tumor cells using a cytotoxic antibody against the podocalyxin-like protein-1, an inhibitor of stearoyl-CoA desaturases or a DNA topoisomerase II inhibitor, etc. Etoposide, a DNA topoisomerase II inhibitor, and the CDK inhibitor purvalanol have been used to minimize the risks of tumor formation by post-transplanted ESCs and iPSCs [345, 346]. Lin et al. reported that the cardiac glycosides digoxin and lanatoside C can kill undifferentiated hESCs [339].

### Important effects of JDP2 on reprogramming-derived CSCs

The activation of the Wnt signaling is critical for maintaining of pluripotency in ESCs [41, 185, 186, 192, 193]. JDP2, has been used as a pluripotency-promoting factor in the reprogramming of cancer cells to reduce their cancerous features. JDP2 can activate or repress various gene transcription actions [185, 361], although it also plays a critical role in malignant transformation. For example, JDP2 can promote cancer cell growth in leukemia and hepatocellular carcinoma [362, 363] but may also be a tumor suppressor in cancer cells [159, 364]. The treatment of gastric cancer cell lines with OCT4 and JDP2 inhibited the tumorigenic function of the cells by switching off BMP7 [195, 365]. The tumor-forming ability of these partially reprogrammed gastric CSC-like cells is reduced in immune-deficient mice, which shows that JDP2 plays a critical role in the reduction of oncogenic potential [185, 189].

Double deficiency of ATF3 and Jdp2 in mice stromal tumors promotes cancer growth [361]. Jdp2 is regarded as a factor that drives reprogramming through the regulation of the Wnt signaling pathway and the suppression of ROS production [188]. Oxygen regulates pluripotent stem cells via Wnt–β-catenin signaling and HIF-1α [188]. Wnt signaling plays a key role in the generation and maintenance of iPSCs [366]. *JDP2* is one of the target genes of the *LEF–TCF* family and is involved in the Wnt signaling pathway [185]. Wang et al. generated iPSC-like cells by introducing *OCT4* and *JDP2* (JO) into gastric cancers for reprogramming [306]. ESC-like colonies were obtained in teratomas of JO-introduced xenografts. The JO-introduced xenografts were smaller and had fewer necrotic and mitotic cells, and a larger nucleus, than the parent cancer xenografts.

The roles of EZH2, HMT, and MLL in the regulation of BMP7 expression have been examined [364, 365]. The findings of this study suggest that HMT inhibitors can be used to prevent MLL and that EZH2 is a potential therapeutic target. The β-catenin–JDP2–RPMT5 complex axis is critical for reestablishing glutathione homeostasis after genotoxic-mediated stress and may be useful in the development of drugs aimed at treating or avoiding inducible resistance to chemotherapy in cancer cells [367]. A combination of factors (Jdp2, Jhdm1b, Mkk6, Glis1, Nanog, Essrb, and Sall4) was reported to be a useful reprogramming complex for efficiently leading mouse embryonic fibroblasts (MEFs) to become chimera-competent iPSCs in xenografts [368]. These findings suggest that the direct reprogramming of stem cells cannot reduce the risk of malignancy itself, and that excluding cancer cells from the microenvironment of stem cells may be crucial for reducing the risk of cancer.

### Other solutions to eliminate the risk of tumorigenesis

Methods of pluripotency reprogramming that do not use genetic material provide another potential strategy for generating safe iPSCs. To date, various molecules that promote cell reprogramming have been reported as substitutes for genetic materials. These small molecules modulate the activities of the enzymes that are involved in the epigenetic modification of genes and may play a crucial role in pluripotency reprogramming [25, 27–30, 369]. These small molecules include the TGFβ inhibitory antagonist SB431542, the MAPK–extracellular signal-regulated kinase inhibitor PD0325901, and the inhibitor of Rho-associated coiled-coil-containing protein kinase thiazovivin (2,4-disubstituted thiazole or TZV). TZV significantly increases the rate of hiPSC reprogramming by up to 200-fold [370]. The combination of *Oct4*, the TGFβ receptor inhibitor A83–01, and the methyltransferase inhibitor AMI-5 increases the reprogramming efficiency of mouse iPSCs, and the repression of ROS increases the efficiency of cell reprogramming [371, 372]. The addition of vitamin C to the culture medium significantly increases the reprogramming efficiency. However, the generation of hiPSCs using small-molecule compounds alone has not been shown to reduce the risk of tumorigenesis significantly. Further investigation of nongenetic compound-guided iPSCs is required to exclude the potential for tumor progression before patient engraftment.

Vitamin C is a candidate for preventing the tumorigenesis caused by hiPSCs because it inhibits the improper self-renewal of human stem cells by increasing histone demethylase activity. Vitanin C has also been applied as an anticancer agent in melanomas [373–376]. The histone demethylases JIhdm1a/1b are the direct downstream molecules of vitamin C. In addition to its antioxidant activity [376], vitamin C was reported to increase the rate of reprogramming of fibroblasts to iPSCs when added to the culture medium [190]. In that study, supplementation with vitamin C decreased p53/p21 levels, which successfully blocked pluripotency reprogramming.

The mutation frequencies in hiPSCs increases with age. Aging is also one of the major risk factors for cancer progression. Therefore, younger donor cells may be used to avoid detrimental mutations in mitochondrial DNA. The reprogramming of somatic cells into iPSCs resets the cellular damage and the stress- and senescence-associated epigenetic marks in vitro, which suggests that the reprogramming technology may be able to induce the rejuvenation of senescent cells [377]. Mosteiro et al. reported that cells reprogrammed in vitro were present next to senescent cells clustered in reprogrammable mice [378]. These senescent cells promote reprogramming through senescence-associated secretory phenotypes, especially via the production of interleukin 6 [379]. The functional crosstalk between reprogramming and senescence has been reported elsewhere [380, 381].

To avoid the risk of point mutations in stem cells, histocompatibility antigen-matched umbilical cord blood-derived iPSCs are useful for ensuring a minimal rate of mutations [382]. Amniotic cells derived from human placental tissues exhibit lower immunogenicity and anti-inflammatory properties than do other cells [383, 384]. The expression of putative immunosuppressors, such as CD59 and CD73, is repressed during the process of reprogramming in amniotic cells [385]. These findings emphasize that long-term-cultured hESCs and hiPSCs show increased growth rates and decreased dependence on the concentration of growth factors and malignant tumor-forming abilities after their engraftment in mice [386]. Carcinoma-derived iPCSCs, which have a higher number of passages, exhibit increased carcinogenic ability compared with those obtained from donor cholangiocellular carcinoma [387].

Other candidate for therapeutic agents includes drugs against the super-enhancers involved in phase separation [388]. In general, the machinery used for epigenetic modification can be altered during transcription initiation, elongation, and termination by involving the transcriptional complex containing polymerase II. Transcriptional regulators such as the mediator MED, coactivator Brd4, splicing factor SRSF2, histone heterochromatin protein 1, and nucleoplasmin 1 may be targets for therapies aimed at modulating chromatin structure during reprogramming and for blocking the development of cancer or other genetic diseases [389]. Hepatocellular carcinomas (HCCs) exhibit distinct promoter hypermethylation patterns. Deletion of C/EBPβ expression using the CRISPR-Cas9 system affects the co-recruitment of BRD4 at enhancers marked with H3K27ac to block the development of HCC [390].

The two mediator kinases, CDK8 and CDK19, may enable transcriptional reprogramming through the super-enhancer family, chromatin looping by CTCF, and cohesion with the transcriptional mediators MED12 and 13, which may be potential drug targets [391]. The valproic acid-mediated inhibition of HDAC and glycogen synthase kinase-3 results in the transcriptional repression of many genes, including the gene that encodes for myristoylated alanine-rich C-kinase substrate 1, which is the Actin-stabilizing protein that is required for the process of the early development of dendritic morphogenesis and synapse maturation [392]. In zebrafish, p300 and Brd4 trigger genome-wide transcriptional network by controlling histone acetylation of the first zygotic genes. This mechanism is crucial for initiation of zygotic development and reproduction [393]. In mammals, these target genes are also potential candidates for drug targets. Stem cell-derived organoids may also be useful for identifying the effects of the microenvironmental niche on cancer development and the reprogramming fates of stem cells [394].

The successful epigenetic reprogramming of primary cancerous cells was recently reported [350]. Pancreatic ductal adenocarcinoma cells were reprogrammed by independent protocols, such as the introduction of *OCT4* together with miRNA of *Mir302*, the episomal vector-encoded *NANOG* and *REX1*, in Yamanaka’s protocol (as a control). These methods yielded efficient reprogramming with reduced tumorigenicity through epigenetic changes, such as downregulation of TET2, SIRT1, disruptor of telomeric silencing 1-like (DOT1L), and T-box 3 (TBX3) and upregulation of TET1. A study of ischemic cardiomyopathy found that DNA methylation and the metabolic pathway were strongly correlated through the EZH2–KLF15 axis [351]. C/EBPβ recruits the DOT1L methyltransferase to open chromatin via methylation of H3K79 in multiple drug-resistance genes [352].

Imprint dysregulation compromises the developmental ability of pluripotent stem cells [353]. The stability of de novo methylation of CpG islands in PSCs is critical for cancer development. Thus, CpG islands and imprinting-control regions are important for the evaluation of development, stemness, and pluripotency [395]. Reprogrammed hiPSCs exhibit greater loss of imprinting compared with ESCs, and the loss of imprinting preexists in their somatic cells of origin. The differently imprinted genes related to the loss of imprinting, especially those of paternal control, are more prone to disruption [396].

Ubiquitin-like with PHD and RING finger domain 1 (Uhrf1) is a hemimethylated DNA-binding protein that interacts with DNMT1 and recruits euchromatic histone–lysine N-methyltransferase 2 to form heterochromatin, together with tripartite motif-containing 28 and HDACs, for DNA methylation. In mouse stem cells, Uhrf1 interacts with the SET domain complex containing 1A/COMPASS, followed by positive regulation of H3K4me3 modification. Uhrf1 maintains bivalent histone marks, such as H3K27me3 and H3K4me3, and particularly those associated with specifications to the neuroectoderm and mesoderm [396]. Tatton-Brown–Rahman syndrome (TBRS) is caused by a mutation in *DNMT3A*, a gene that is also associated with Sotos syndrome, which is caused by haploinsufficiency of *NSD1*, an HMT that catalyzes the demethylation of histone H3 at K36 (H3K36m22). In the mouse, NSD1-mediated H3K36me2 methylation is induced by the recruitment of DNMT3A and is crucial for the maintenance of DNA methylation at intergenic regions. The binding of DNMT3A to H3K36me2 can be inhibited by a missense mutation associated with TBRS, which suggests that trans-chromatin regulatory control is critical for human neoplastic and developmental growth [397].

## Conclusion

Genetic or epigenetic alterations in proteins or microenvironmental niches might promote the initiation or progression of carcinogenesis in some cells. Further steps should be taken to provide effective anticancer systems for the therapeutic application of reprogramming-guided human stem cells. One intriguing technique is the use of a CRISPR-Cas-derived vector to remove the targeted region of epigenetic barriers to identify the effects of transcriptional reprogramming. Targeting of dCAS9-VP64 to the *Sox1* promoter produces strict transcript and protein upregulation in neural progenitor cells. The removal of DNA methylation by dCas9-Tet1 increases the proportion of cells with activating master key transcription factors for abrogating the barriers of cell fate [398]. The single-cell sequencing technique is also critical for defining cell fate and the decision toward differentiation.

The ascorbic acid plus 2i and Dot1l inhibitor drugs can rapidly affect the conversion of MEFs to iPSCs. The stemness gene *Nanog* appears in a subcluster with genes such as those encoding the epithelial cell adhesion molecule (*Epcam*), Sal-like protein 4 (*Sall4*), and *thymine DNA glycosylase genes (Tdg). The Tdg tandem duplicate 1 (Tdg1*) and *Oct4* cluster with *Zfp42,* and *Sox2* clusters with the undifferentiated embryonic cell transcription factor 1 (*Utf1*) and the developmental pluripotency-associated protein 5A (*Dppa5a*). Sustained coexpression of *Epcam*, *Nanog*, and *Sox2* with other genes is also required for progression of MEFs toward iPSCs. The genes for Ets homologous factor (*Ehf*), *pleckstrin* homology-like domain family A member 2 (*Phlda2*), and eukaryotic initiation factor 4A-I (*Eif4a1*) also play critical roles in robust iPSC generation.

Regulatory network analyses allow the search for new networks of signaling, such as signaling inhibition by 2i, and their role in repressing somatic expression. Such analyses also allow the comparison of the actions of the epigenetic modifier ascorbic acid and a Dot1l inhibitor for pluripotent gene activation [399]. In one study, human iPSC-derived neurospheres were transferred into nonobese diabetic-severe combined immune-deficient mice, to treat and cure a spinal cord injury without any tumor generation [349]. These grafted hiPSC-NSs survived, migrated, and differentiated into functional neurons. However, the direct application of undifferentiated iPSCs or hPSCs to patients has not been reported and further research and advances are needed to generate transplantable stem cells or organoids that can be applied to patients in the near future.

Collectively, the data discussed in this review show that the characteristics of pluripotency can inhibit the features of the cancer phenotype, restore differentiation potential, and change the expression of the indicated cancer-related genes through epigenetic modifications, chromatin organization, and metabolism reprogramming (Table 2). Therefore, the targeting of these epigenetic alterations may provide effective approaches for inhibiting the tumorigenic capability of CSCs in the future. Further study is required to provide further understanding of the molecular machineries underlying the reprogramming of cancer cells and the development of novel therapies for the regenerative reprogramming of human cancer cells and their derived organoids.

## Data Availability

Not applicable.

## Abbreviations

BMP7: Bone morphogenetic protein 7
CNVs: Copy number variations
CSCs: Cancer stem cell
DNMT: DNA methyltransferase
EMT: Epithelial mesenchymal transition
ESCs: Embryonic stem cells
EZH2: Enhancer of zesta
HDAC: Histone deacetylase
hESCs: Human embryonic stem cells
hiPSCs: Human induced pluripotent stem cells
iPSCs: Induced pluripotent stem cells
JDP2: Jun dimerization protein 2
miRNA: MicroRNA
OSKM: Oct4, Sox2, Klf4 and c-Myc
OSNL: Oct4, Sox2, Nanog, and Lin28
PGE2: Prostaglandin E2
PRC: Polycomb repressive complex
PSC: Pluripotent stem cells
ROS: Reactive oxygen species
SCD: stearoyl-CoA desaturase
TERT: Telomerase reverse transcriptase
TET: Ten-eleven translocation protein
TGFβ: Transforming growth factor β
